The article "Image Processing Technology in Remote Monitoring and Intelligent Medical System" was published in 2021. Journal: J Healthc Eng.

# Image Processing Technology in Remote Monitoring and Intelligent Medical System

**DOI:** 10.1155/2021/6549891

**Published:** 2021-11-22

**Authors:** Kongjun Bao, Yaoxi Bao

**Affiliations:** ^1^Engineering Training Centre, Zhengzhou University of Light Industry, Zhengzhou 450000, China; ^2^Outpatient Department of Xicheng Branch, Luohe Central Hospital, Luohe 462400, China

## Abstract

In order to study the application of image processing technology in remote monitoring and intelligent medical systems, the principle and implementation method of a remote intelligent image monitoring system based on virtual local area network is proposed; this method analyzes the key technologies to be considered in the remote realization of image monitoring, adopts advanced digital image compression coding and decoding technology and digital image transmission technology, and applies intelligent image processing and recognition technology to display, adjust, and track images; it overcomes the defects that the general monitoring system requires excessive intervention by monitoring personnel and low intelligence. After verification, the experimental results show that the proposed model can accurately and efficiently segment nonoverlapping cervical cell images, and compared with other existing models, this model has both higher segmentation accuracy and faster calculation speed. The application of multicast is still only in the laboratory or small local area network; with the further development of network technology, its application prospects will be very broad.

## 1. Introduction

Images are not strange to us. They are obtained by observing the objective world in different forms and methods with various observing systems, an entity that can directly or indirectly act on the human eye and thereby produce visual perception. Human vision is an observation system; the image obtained through it is the image formed by the objective scene in people's mind. Normal images are simulated images; that is, the information on the image is a continuously changing analog quantity [1]. For example, the objects on a black and white grayscale photo are reflected by the light intensity of each point on the photo, and the light intensity on the photo is a continuously changing quantity; in other words, within a certain range, any value of light intensity may appear. Therefore, computer image processing is often referred to as digital image processing. Image processing technology began in the 1950s; in 1964, the US Jet Propulsion Experiment (J.PL) used a computer to process a large number of photos of the moon sent back from the spacecraft to obtain clear and realistic images; this is an important milestone in the development of this technology. Since then, image processing technology has been widely used in space research [2]. In the early 1970s, due to a lot of research and application, digital image processing has its own technical characteristics and formed a relatively complete discipline system, so as to become an independent new discipline. The process of image processing and analysis usually includes fetching data from a capture card with frame memory to computer memory, processing the image data in the memory, and sending the data back to the image frame memory in three steps; the capture card directly uses the internal memory, and you only need to exchange data with the memory (some use software algorithms, but it is not common and the effect is not necessarily good). An important fact in image processing and analysis is that special solutions are needed for special problems; to solve specific problems, specific in-depth research and analysis are needed. Research has shown that Aparna and Kishore first proposed the concept of end-to-end fully convolutional network (FCN) based on the idea of semantic segmentation, performed convolution processing on the entire input image, and learnt high-dimensional abstract information, through deconvolution processing to obtain the segmentation output of different kinds of pixels [3]. Zhu et al. used the FCN framework to study the segmentation of MRI images of multiple sclerosis lesions; although the data set used for segmentation is small, a DSC value of 68.4 was still obtained [4]. Kario further used this network framework to segment MRI images of normal human tissues and tested the influence of single-mode and multimodal input on the network, showing that the model pump obtains richer high-dimensional information from multimodal input [5].

### 1.1. System Overview

The remote intelligent monitoring system is mainly composed of communication links, the monitoring center, and multiple monitoring remotes. The communication link refers to the transmission channel and related equipment used. The communication network supports various methods such as PSTN, DDN, ISDN, LAN/WAN, EI dedicated line, microwave, wireless spread spectrum, or satellite line. Data transmission channels are established between communication centers. The peripheral equipment used by the remote monitoring system of the monitoring system includes the remote monitoring host, alarm collector, temperature and humidity sensor, screen splitter, camera, pan-tilt and variable lens, microphone, and speaker [6–8]. The monitoring center has network equipment such as TV walls, disk arrays, servers, switches, and routers, as shown in Figure 1.

The monitoring system adopts advanced digital image compression coding and decoding technology, digital image transmission technology, apply intelligent image processing, and recognition technology to the display of images and the tracking of the monitoring site and provides a voice channel and a variety of alarms; the linkage function can provide a variety of line interfaces [9]. The system can set different schemes according to the actual needs of users; the good openness makes this system have a broad application market, and its system structure block diagram is shown in Figure 2.

The back-end monitoring equipment is composed of a web video monitoring server and a number of remote control computers, web video surveillance server includes video surveillance server and web server, and the two servers can be installed on the same or different hosts. The remote subcontrol computer can be the host in the local area network, and it can also be a host that dials up the Internet through the model. Data from different monitoring sites are input to the video surveillance server through the communication device; they are forwarded to the network by the monitoring server and adopted the technology that combines point-to-point transmission and multicast. In this way, the subcontrollers on the local area network and the wide area network can be monitored at the same time through the browser [10]. Each user can monitor multiple front ends at the same time, that is, “point to many points.” Different users can also monitor the same front end at the same time, that is, “multiple points to one point,” and have great flexibility. In addition to translating pronunciation video data, the web video surveillance server also completes the management of the entire monitoring system, control and remote subcontrol management, and control transmission.

### 1.2. System Tracking Implementation

Image tracking must complete the following tasks. (1) Search, that is, in the observed scene image: the area where the image target exists is searched; (2) detection, segmentation, and recognition; and (3) the target point and its whereabouts, that is, the point representing the target position are determined on the image target, and its position is determined, and the trajectory of the image target over time is given. Image processing: in order to realize the tracking function of the system, multithreaded programming is used in the remote monitoring and monitoring center [11–13]. One thread is used for image capture and compression, and one thread is used for real-time processing of images. The image processing module processes the collected images regularly, obtains the brightness, and focuses on information of the image; if it does not meet the requirements, the camera's aperture, brightness, and focal length are adjusted by issuing control commands and the quality of the captured image is automatically protected (you can also manually adjust the camera's iris, brightness, and focal length). The automatic adjustment module of the image can meet the screen requirements of the monitoring image of multiple monitoring points at the same time and avoid adjustments and omissions of monitoring personnel [14]. When the system is in the automatic tracking state, it can detect moving objects, obtain the edge, and shape characteristics of moving objects, and obtain the movement state of the moving object, through a certain tracking algorithm.

### 1.3. Image Compression

Video image compression is divided into lossless compression and lossy compression. Lossless compression means that when playing back compressed files, the original data can be restored accurately. This is often used to compress data files, such as ZIP files. The commonly used algorithm for lossless compression is the number counting method, it defines a series of the same color as two parameters of color and quantity, and this reduces the space occupied by the same color. It can be seen that this compression algorithm is very useful when compressing black and white pictures; however, it is not practical to compress active color images, it is too much affected by the complexity of the image, resulting in too low compression rate, and it is difficult to exceed the compression rate of 3 : l [15].

### 1.4. Image Processing Technology of Remote Intelligent Image Monitoring System

If the target and background in the image have different grayscale sets: target gray set and background gray set and two grayscale sets can be divided by a grayscale closed value *T*, for example, the height set is the target gray level set, in this way, we can divide the target area and the background area in the image with the method of interpreting the grayscale [16]. This method is called grayscale value segmentation.

This method is particularly useful for segmenting objects and backgrounds in a scene image where there is a strong contrast between the object and the background, especially the gray distribution inside the object is uniform and the background is also uniform. If the difference between the object and the background lies in certain features rather than grayscale features, then you should first use these feature differences to identify the object and the background and convert it into the difference in grayscale; under the condition of the aforementioned closed value segmentation, the closed value segmentation is performed again. Under this transformation, the use of audible value segmentation techniques may also be very effective. Then, the image area and its shape *f*_(*T*)_(*x*, *y*) after segmentation according to the above method can be expressed by the following formula:

(1) $$\begin{array}{c} f_{\left(T\right)}\left(x,y\right)=\left\{\begin{array}{cc} 1, & f\left(x,y\right)\geq T,\\ 0, & f\left(x,y\right)<T, \end{array}\right\},\\ g\left(i,j\right)=\left\{\begin{array}{cc} g_{0}, & f\left(i,j\right)\leq T_{0},\\ g_{1}, & T_{0}<f\left(i,j\right)\leq T_{1},\\ g_{n}, & f\left(i,j\right)>T_{n-1}, \end{array}\right\}, \end{array}$$

where *f*(*i*, *j*) is the gray value of the original image pixel; *g*(*i*, *j*) is the output result of pixels on the image after region segmentation processing; *g*_0_,  *g*_1_,  and *g*_*n*_ are the treated background *s*_0_, the output value of pixels in area *s*_1_, area *s*_2_, and area *s*_*n*_ or some kind of mark. After each point of the image is processed by the above gray threshold method, each meaningful area is separated from the image background.

In simple images, there are often only two areas, the background and a meaningful part; at this time, only a threshold value needs to be set, can complete the segmentation process, and form a binary image with only two gray values. Sometimes, the same type of meaningful area appears multiple times in the image, they have the same characteristics, belonging to the same kind of scenery, and at this time, an area is composed of multiple subareas [17].

#### 1.4.1. The Maximum Variance Automatic Cut-Off Method

The shape of the image grayscale histogram is changeable. It has double peaks, but no obvious troughs and the double peaks. Its troughs are not obvious, and it is often difficult to determine the area ratio of the two regions; at this time, using the maximum variance automatic leap method can often get a more satisfactory result.

The relationship between the average gray value of the entire image and the average gray value of area 1 and area 2 is as follows:

(2) $$\begin{array}{c} \mu =\mu_{1}\theta_{1}+\mu_{2}\theta_{2}. \end{array}$$

The same area often has similar grayscale characteristics, and the old area of each area is obviously different in grayscale; when the grayscale difference between the two regions separated by the threshold *t* is large, the average grayscale of the two regions, the difference between *μ*_2_ and the average gray level *μ*_1_ of the entire image is also large; the variance between regions is an effective parameter to describe this difference, and its expression is as follows:

(3) $$\begin{array}{c} \sigma_{B}^{2}\left(t\right)=\theta_{1}{\left(\mu_{1}-\mu \right)}^{2}+\theta_{2}{\left(\mu_{2}-\mu \right)}^{2}. \end{array}$$

### 1.5. Image Segmentation Based on Edge Extraction

Image edges are very useful for image recognition and computer analysis. The edge can outline the target object and make it clear to the observer. The edge contains rich internal information (such as direction, step property, and shape); it is one of the important image features in image recognition [3]. Essentially, the edge of an image is a reflection of the discontinuity of the local characteristics of the image (grayscale mutation, color mutation, texture structure mutation, and so on); it marks the end of one area and the beginning of another.

Edge extraction first detects the discontinuity of the local characteristics of the image and then connects these discontinuous edge pixels to form a complete boundary. The characteristic of the edge is that the pixels along the edge change smoothly and the pixels perpendicular to the edge change drastically. So, in this sense, the algorithm for edge extraction is a mathematical operator that detects edge pixels that meet the edge characteristics. The basic edge detection operators include gradient operator, Robert gradient operator, Sobel operator, Laplacian operator, Kirsch operator, and Rosenfeld operator. The classic edge extraction is based on the original image; for each pixel of the image, the change of gray level in a certain area of it is examined and the first-order or second-order directional derivative change rule of the neighboring domain of the edge is used to detect the edge.

For the common edges in Figure 3, the gray level changes may be either step-shaped or pulse-shaped [18].

## 2. Materials and Methods

In the experiment of partial cytoplasm overlapping cervical cells, to test the segmentation problem of “partially overlapping” cervical cell color image, test for segmentation of “true overlap” cervical cell EDF images, the data sets used are in 2014 and 2015, two datasets released by the overlapping cervical cell image segmentation challenge constructed by the University of Adelaide. Here, we abbreviate the two overlapping cervical cell challenge data sets as ISBI2014 overlapping cell data set and ISBI2015 overlapping cell data set. The ISBI2014 overlapping cell data set contains 945 synthetic overlapping cervical cell images with a size of 512 × 512; among them, 45 are training pictures and 900 are test pictures. The ISBI2015 overlapping cell data set contains 17 real cervical multicell pictures with a size of 1024 × 1024; among them, 8 can be used as training pictures and 9 can be used as test pictures.

### 2.1. Evaluation Index

The indicators used to evaluate the “true overlap” segmentation results in the ISBI data set include ZSI, object-based false negative rate (FNo), positive samples based on pixel-based correct classification (pixel-based true positive rate, TPp), and pixel-based false positive rate (FPp). According to the explanation on the overlap segmentation index on the ISBI Challenge website, a “good” segmentation means that the average ZSI of the segmented region results is >0.7; the larger the ZSI value, the better the segmentation effect. FNo is the proportion of errors calculated in cells when ZS I ≤ 0.7 [19].

## 3. Results and Discussion

### 3.1. Image Segmentation Results and Analysis

Due to the use of Herlev and Guan two data sets, therefore, the evaluation of the segmentation results of some cytoplasmic overlapping cervical cells is divided into two parts, as shown in Table 1.

It can be seen from Table 1 that from the ZSI indicators of the four methods, all of them are greater than 0.7, indicating that the four methods are all “good” segmentation, but the ZSI average value of this model is the largest at 0.83; it proves that the improved super-pixel K-means++ model proposed in this chapter is better than the other three models. For such methods based on super-pixels, the same segmentation method on the Herlev data set is slightly better than the result on the Guan data set. The pixel-based method is slightly better than the result of the Herlev data set on the Guan data set. The reasons for the analysis to produce such results are the image resolution of the Herlev dataset is higher than that of the Guan dataset, and because the super-pixel oversegmentation algorithm can better capture the target edge in high-quality images, therefore, the segmentation effect of methods based on super-pixels on the Herlev dataset is better.

Aiming at the segmentation problem of “true overlap” cervical multicell EDF images, a combined segmentation model based on graph cut and Voronoi diagram is proposed. The model first uses the graph cut method to distinguish the image background and the cell cluster area, then the Voronoi diagram algorithm is used to roughly divide the cell clusters to get the rough contour of each cell, then the cell overlapping area is further compensated and segmented, and finally the coarse division cells and the overlapping compensation area are combined to obtain complete cells. The experimental results of this segmentation model on the data sets of the two overlapping cervical cell segmentation contests in 2014 and 2015 show that the segmentation effect of this model is good, the effect is equivalent to the existing excellent segmentation model for dealing with such problems, and the lack of training data is an important advantage of this model. There are also some problems with this method. The correct detection of cell nuclei is highly dependent, and the segmentation effect needs to be further improved. Future work should focus on two aspects: one is to continuously explore new algorithms to improve the accuracy of cell nucleus detection and segmentation and the second is to use more detailed cell prior shapes to improve the accuracy of overlapping regions segmentation.

## 4. Conclusions

This thesis is based on an actual video communication subject; many practical and advanced image processing and programming techniques are used; and in the actual design of the remote image monitoring system, using object-oriented design ideas and distributed processing implementation methods, the overall structure of the system and the proposed solutions are relatively leading in China. It realizes the network and intelligence of remote image monitoring through adopting intelligent control technology in tracking control. The overall system structure and key technologies of the intelligent remote monitoring system are introduced, and the new application and specific implementation of multicast technology in the remote monitoring image transmission of distributed manufacturing systems are discussed. The problem of multimachine monitoring is also solved. However, the implementation of the current multicast routing protocol is still in the experimental stage mainly because the router connected to the network does not support the forwarding of multicast data. The application of multicast is still only in the laboratory or small local area network, with the further development of network technology; its application prospects will be very broad.

## Figures and Tables

**Figure 1:** Front-end equipment.

**Figure 2:** Block diagram of the intelligent remote monitoring system.

**Figure 3:** Concepts of first-order difference and second-order difference of common edges.

**Table 1:** “Partially overlapping” cell image quality segmentation results of Herlev data set.

Segmentation method	*μ*ZSI ± *σ*ZSI
Based on pixel K-means	0.75 ± 0.23
Based on pixel spatial K-means	0.76 ± 0.15
Based on the super-pixel EM algorithm	0.81 ± 0.13
Improved model of super-pixel K-means++	0.83 ± 0.16

## Data Availability

The data used to support the findings of this study are available from the corresponding author upon request.
